The article "Analysis of the effects of in-situ chemical oxidation on microbial activity using Pseudomonas putidaF1" was published in 2021. Journal: Heliyon.

# Analysis of the effects of *in-situ* chemical oxidation on microbial activity using *Pseudomonas putidaF1*

**DOI:** 10.1016/j.heliyon.2021.e08665

**Published:** 2021-12-23

**Authors:** Mohan B. Dangi, Michael A. Urynowicz, Christopher L. Schultz, Samir Budhathoki, Sadikshya R. Dangi

**Affiliations:** a Department of Geography and City & Regional Planning, California State University, Fresno, CA, 93740, USA; b Department of Civil & Architectural Engineering, University of Wyoming, Laramie, WY, 82071, USA; c Trihydro Corporation, Soldotna, AK, 99669, USA; d US Department of Agriculture, Agriculture Research Service, Northern Plains Agricultural Research Laboratory, Sidney, MT, 59270, USA

**Keywords:** *In-situ* chemical oxidation, Biometer study, *Pseudomonas putida F1*, Bioavailable carbon, Toluene, Catalase

## Abstract

*In-situ* chemical oxidation is an effective groundwater remediation approach for delivering oxidants to the subsurface environment where various contaminants of concern, natural organic matter, and other reduced species within the soil consume the oxidants. The addition of these oxidants alters microbial activity changing the physical and chemical structure of the soil. This paper studied the effects of chemical oxidation on microbial activity with and without toluene. Several oxidants were used as part of the study: sodium percarbonate, hydrogen peroxide, potassium permanganate, and sodium persulfate evaluated at low, medium, and high concentrations. A series of biometer experiments seeded with microbe *Pseudomonas putida F1* and soil sample and aqueous toluene solution for each oxidant was monitored by CO_2_ production as a function of incubation days to evaluate the effects of oxidation on the microbial activity. Of the oxidants tested, permanganate oxidation resulted in the highest increase in microbial activity post oxidation based on CO_2_ production both with and without the addition of toluene. The other oxidants exhibited a direct correlation between oxidant concentration and the change in permanganate chemical oxidant demand of the soil. However, there was no correlation between oxidant concentration and microbial activity. Each of the oxidants was shown to increase CO_2_ yield except for sodium percarbonate, which had an adverse effect on microbial activity. It is likely that the increased microbial activity associated with permanganate oxidation was the result of chemical reactions between the oxidant and natural organic matter in the soil.

## 1 Introduction

In water and wastewater systems, chemical oxidation has been used for over three decades to remove recalcitrant organic contaminants and petroleum hydrocarbons (Devi et al., 2016; Liu et al., 2014; Sutton et al., 2011). *In-situ* chemical oxidation (ISCO) is a widely used technology for the remediation of soil and groundwater at hazardous waste sites (Devi et al., 2016; Liang and Su, 2009; Tsitonaki et al., 2010). It is considered an effective, low cost, fast, and relatively low maintenance remediation technique for the destruction and removal of some non-aqueous phase liquids, which can be challenging to remediate using other methods (Khodaveisi et al., 2011; Sutton et al., 2011; Romero et al., 2009).

Several strong oxidants can be used in the ISCO process; however, this paper focuses on permanganate (MnO_4_^-^), persulfate (S_2_O_8_^-^), hydrogen peroxide (H_2_O_2_), and percarbonate (CO3·1.5 H2O2^2-^). Table 1 provides the list of chemicals studied in the paper (Huling and Pivetz, 2002; Khodaveisi et al., 2011; Miao et al., 2015a, 2015b, and 2015c). Permanganate is available as a salt (KMnO4 and NaMnO4) and has been widely used as an ISCO oxidant for the remediation of contaminated soil and groundwater systems (King et al., 2021; Khodaveisi et al., 2011; Li and Schwartz, 2004). Previous studies (Liu et al., 2014; Waldemer and Tratnyek, 2006) have suggested that permanganate is less powerful than other oxidative species but reacts quickly with specific contaminants including chlorinated ethenes. It also produces manganese oxide (MnOx) solids, which can clog soil pores and reduce oxidant transport in the subsurface.

**Table 1:** The list of chemicals studied in the research.

Name of the chemicals	Doses	Concentration (g/L)
Potassium permanganate (Aldrich)	Low	0.50
	Medium	1.00
	High	2.00
Hydrogen peroxide (Mallinckrodt)	Low	0.46
	Medium	0.93
	High	1.87
Sodium persulfate (Aldrich)	Low	0.41
	Medium	0.83
	High	1.66
Sodium percarbonate (Aldrich)	Low	1.56
	Medium	3.13
	High	6.25

Hydrogen peroxide is one of the most used oxidants for the remediation of organic contaminants in wastewater systems (Devi et al., 2016; Khodaveisi et al., 2011). It can exhibit both oxidant and reductant properties and can also be used as an oxygen source (Devi et al., 2016). A study (Xu and Li, 2010) demonstrated that the oxidation potential of H_2_O_2_ is higher than that of molecular oxygen, and it is effective over a wide range of reaction conditions (acidic to alkaline). Under aerobic conditions, hydrogen peroxide can decompose into molecular oxygen (Interscience, 1910). When catalyzed with ferrous ion, hydrogen peroxide can produce Fenton's reagent, forming a hydroxyl radical (OH^−^) and hydroxide ion in the process. Fenton's reagent is an even stronger oxidizing agent than hydrogen peroxide, capable of oxidizing a wide range of organic contaminants (Atalay and Ersöz, 2016). Fenton's reagent has been shown to be even more efficient at removing chemical oxidant demand (COD) when combined with ozone (Fe^2+^/H_2_O_2_/O_3_) as a part of the advanced oxidation process (Buthiyappan et al., 2016; Cuerda-Correa et al., 2020; Hamidi and Salem, 2015). However, high levels have been shown to be toxic to microorganisms (Pardieck et al., 1992).

Like permanganate, persulfate is available as sodium persulfate (Na_2_S_2_O_8_). Persulfate degrades into sulfate which, according to the United States Environmental Protection Agency (USEPA), has a secondary maximum contaminant level (MCL) of 250 mg/L, as compared to manganese which has a secondary MCL of 0.05 mg/L. Like permanganate, persulfate has also not been shown to significantly hinder microbial activity (Khodaveisi et al., 2011).

Percarbonate is available as sodium percarbonate (2Na_2_CO_3_.3H_2_O_2_) and has become more popular as an alternative for conventional H_2_O_2_ (Ma et al., 2018). Recent studies suggest that sodium percarbonate is effective in degrading organic pollutants both in soil (Apul et al., 2016; Cajal-Mariñosa et al., 2012; Viisimaa and Goi, 2014) and water (Cui et al., 2017; Danish et al., 2017; Fu et al., 2015; Miao et al., 2015a; Miao et al., 2015c) over a wider range of pH as compared to that of H_2_O_2_. Sodium percarbonate is also more stable than H_2_O_2_; however, despite these advantages, relatively few studies are on the effectiveness of sodium percarbonate for degrading the organic contaminants in the subsurface environment (Ma et al., 2018).

Each of these oxidants reacts differently with the target (i.e., contaminants of concern), and non-target (i.e., natural organic matter (NOM) and other reduced species) compounds (Urynowicz, 2007) and it has been demonstrated that non-target compounds can exert a natural oxidant demand (NOD) orders of magnitude greater than that of the target compounds. However, this demand goes unreported for oxidants other than permanganate, primarily due to difficulties regarding analyses. This study used biometers (seeded with *Pseudomonas putida F1* with and without toluene) with various oxidants added at different concentrations (low, medium, and high) to evaluate the effects of in-situ chemical oxidation on microbial activity. This effect was monitored by establishing the direct correlation between microbial activity and the production of carbon dioxide gas over time. The post-oxidation biometers were used to determine if ISCO with the various oxidants altered the soil in ways that increased or decreased microbial activity. Previous studies were also performed using pre-and post-oxidation biometers to further assess the changes in microbial activity (Bolade et al., 2021; Huang et al., 2018).

## 2 Materials and methods

The chemicals used were reagent grade potassium permanganate (Aldrich), sodium percarbonate (Aldrich), hydrogen peroxide (Mallinckrodt), sodium persulfate (Aldrich), monosodium potassium phosphate (Fisher), dibasic potassium phosphate (Fisher), glycerol (Fisher), 1 N barium chloride (Fisher), phosphate-buffered saline, and phenolphthalein pH indicator. Permanganate chemical oxidant demand (PCOD) removal was determined to evaluate the amount of NOD of the soil following chemical oxidation with permanganate, hydrogen peroxide, sodium persulfate, and percarbonate using a modified test developed by Xu and Thomson (2008). Low (0.5 g/L), medium (1 g/L), and high (2 g/L) KMnO4 concentrations were selected based on the results from previous studies (Urynowicz et al., 2008). Equivalent concentrations for the other three oxidants were established based on each oxidant's oxidation potential (See Table 2).

**Table 2:** Experimental conditions for the natural oxidant demand study.

Oxidant	Oxidation potential	Initial oxidant concentration (g/L)
Permanganate	1.67	0.50
Permanganate		1.00
Permanganate		2.00
Hydrogen peroxide	1.78	0.46
Hydrogen peroxide		0.93
Hydrogen peroxide		1.87
Persulfate	2.01	0.41
Persulfate		0.83
Persulfate		1.66
Percarbonate 30% H_2_O_2_	0.53	1.56
Percarbonate 30% H_2_O_2_		3.13
Percarbonate 30% H_2_O_2_		6.25

This experiment prepared a 0.5 M Sorensen phosphate buffer using 0.5 M solutions of sodium phosphate dibasic and potassium phosphate monobasic (Hyat, 1989). The soil used was prepared by the following procedure. Soil samples from several contaminated sites were placed in an evaporative oven at 105 °C for 24 h to remove the moisture and volatile organic contaminants. The dried soil samples were homogenized using a mortar and pestle and mixed to form a composite soil sample (Urynowicz et al., 2008). Deionized water was used and prepared by distillation and filtration with a Barnstead distiller and nano-pure filtration system. The Haas Broth was prepared using the following chemicals: magnesium sulfate (Aldrich), calcium chloride (Fisher), monopotassium phosphate (Sigma), diammonium hydrogen phosphate (Aldrich), potassium nitrate (Aldrich), and ferric chloride (Fisher). This approach prepared both nutrient broth (Difco), nutrient agar plates, and aqueous toluene by adding excess pure phase toluene (Fisher) to deionized water allowing dissolution to occur over time in a sealed amber glass bottle fitted with a 2 ml bottle-top dispenser. Hydrochloric acid (0.1 M) and potassium hydroxide (0.1 M) were purchased from Baker Chemical and diluted to 0.05 M. This project purchased a pure culture of *Pseudomonas putida F1* (ATCC strain 700007) from ATCC: The Global Bioresource Center (ATCC, Manassas, VA, USA) and was shipped freeze-dried (Abuhamed et al., 2004; Huang et al., 2013a, 2013b, 2018).

*Pseudomonas putida* strains exhibit a high degree of biodegradation capacity (Pal and Giri, 2021) and *Pseudomonas putida F1* has been shown to degrade various BTEX compounds including toluene as a primary substrate (Bordel et al., 2007; Huang et al., 2013a, 2013b, 2018; Chicca et al., 2020). The bacteria's metabolic pathways have a higher degree of convergence, and many of its induced enzymes are nonspecific similar to other pseudomonads (Reardon et al., 2000). *Pseudomonas putida F1* is not pathogenic to plants and animals and can be characterized as one of the best hydrocarbon-degrading bacteria capable of metabolizing various hydrocarbons as a sole carbon source (Robledo-Ortíz et al., 2011; Timmis 2002). The bacterium is aerobic and capable of growing on both nutrient broth and nutrient agar at 30 °C, making it easy to work with and grow in a laboratory (Diaz et al., 2008).

The biometer tests were performed with soil samples previously treated with the various oxidants. The soil samples were oxidized by adding 3 g of soil and 30 mL of each oxidant at low, medium, and high concentrations and tumbled, using a Barnstead lab-quake tumbler for two weeks. The samples were then added to biometer flasks both with and without the addition of an aqueous toluene solution. The study aimed to correlate the microbial degradation of toluene as a sole carbon substrate following oxidant treatment with the rate of CO_2_ production (μmoles).

### 2.1 Bacterial growth experiments

The experiments used a *Pseudomonas putida F1* culture to inoculate a beaker of sterile nutrient broth. The nutrient broth and nutrient agar solutions were sterilized by autoclaving at 120 °C for 20 min. The inoculated broth was streaked for isolation to ensure a pure culture and then grown in a glycerol and nutrient broth solution, preserved in a nitrogen freezer at -70 °C for future use.

Once the bacterium had been successfully grown in nutrient broth and agar, the experiment determined bacterial growth kinetics and populations to establish an effective and consistent inoculation process. The first step was developing a consistent inoculation procedure that would minimize the lag time and produce a sufficient cell count. A flask containing 150 mL of nutrient broth was inoculated with a single pure culture collected from a nutrient agar plate. This sample was grown in an incubator for fifteen hours, allowing the bacteria to progress through the lag phase into the exponential growth phase. Then, three other flasks containing 150 mL of nutrient broth were inoculated using one milliliter of the freshly grown bacteria. Optical density measurements were taken every two hours with a spectrophotometer at 600 ηm. The samples were also measured periodically using plate counts to determine the number of viable cells at points along the growth curve.

The optimal time for the bacteria used to inoculate the biometers was determined to be 30 h (the transition between exponential growth and plateau phases) when the maximum number of viable cells was present (3×10^12^ per mL). It also provided the most consistent results from batch to batch. The following procedure was used to ensure that the biometers were inoculated consistently for all experiments while minimizing additional carbon added to the system. First, the bacteria were grown and isolated on nutrient agar plates. A single pure culture of the organism was then added to a 150 ml beaker of sterile nutrient broth and grown for 15 h at 30 °C. Then, 1 ml of this bacterial culture was added to 150 ml of clean nutrient broth (BD Difco TM, Franklin Lakes, New Jersey, USA) and grown for approximately 30 h to an optical density reading of 1.5 at 600 ηm. An aliquot of 20 ml of cells was washed by centrifuging at 4000 rpm. The experiment finally decanted the excess nutrient broth. The cells were re-suspended in a solution of phosphate-buffered saline to remove residual carbon from the unused Haas Broth to produce a low residual carbon inoculum.

### 2.2 Biometer experiments

This experiment used a series of biometer flasks to determine the amount of CO_2_ produced by the microorganisms as a function of time. See Figure 1. The CO_2_ gas was then trapped when it dissolved into the potassium hydroxide (KOH) solution (10 ml of 0.05 M) to fill the sidearm. Pritchard et al. (1992) provide detailed diagrams for the typical biometer setup. Titration was performed on the KOH solution using 0.05 M hydrochloric acid to determine the amount of CO_2_ produced (Pramer and Bartha, 1965; Pritchard et al., 1992; Mariano et al., 2008). Table 3 shows the detailed experimental conditions.

**Figure 1:** Schematic layout of biometer flask.

**Table 3:** Experimental conditions.

Section	Experimental condition	Oxidized soil and slurry (6 g and 60 ml)	Unoxidized soil (6 g)	Toluene addition (8 ml)	Hass broth (60 ml)	Microbial inoculum (1 ml)	Sorenson phosphate buffer (6 ml)
4.1	Control		x	x	x	x	
	Control		x		x	x	
	Control			x	x	x	
	Control				x	x	
	Control				x		
4.2	Potassium permanganate^1^	x		x		x	x
	Potassium permanganate^1^	x				x	x
4.3	Hydrogen peroxide^1^	x		x		x	x
	Hydrogen peroxide^1^	x				x	x
4.4	Sodium persulfate^1^	x		x		x	x
	Sodium persulfate^1^	x				x	x
4.5	Sodium percarbonate^1^	x		x		x	x
	Sodium percarbonate^1^	x				x	x
	Sodium percarbonate^1^	x					x

1 Each experiment was conducted for low, medium, and high concentrations, 0.5 g/L, 1 g/L, and 2 g/L as KMnO_4_.

Sorenson phosphate buffer (Bellco Glass, Inc., Vineland, New Jersey, USA) was used for the experiments as phosphate buffers are found in living systems and are typically non-toxic to cell growth (Hyat, 1989). This experiment added six milliliters of the Sorenson phosphate buffer solution to the I-Chem bottles before transferring the soil water matrix to the biometer flasks. This amount was determined as the minimum amount of buffer required to keep each oxidized soil and water solution between a pH of 7 and 8. The available oxygen within the biometer flasks was determined to ensure that oxygen was not limiting. Based on stoichiometry, coupled with the assumptions that the system's volume is 300 ml and the oxygen in the liquid sample is negligible, the system has 49 mg of oxygen available in the headspace. Biometer tests produced 700 mmol of CO_2_ (at the most), equal to 29 mg of oxygen consumed or roughly 60% of the available oxygen in the closed biometer flask. It was sufficient oxygen for the test and confirmed that oxygen was not a limiting factor.

The following steps were performed for each microcosm experiment. First, the media solution (Table 1) was added to the 250 mL biometer flask. Then an aqueous phase toluene solution (8 ml) was added to the biometer flasks immediately before sealing. The toluene concentration of the solution was 115 ± 25 mg/L. Experiments used this same solution of toluene and water for all additions. The 115 mg/L toluene solution can produce 63 ± 8 μmol of CO_2_ when completely degraded to CO_2_ by the microorganisms. See Eq. (1). The biometers were then sealed with rubber stoppers, and 10 mL of 0.05 N KOH solution was injected into the sidearm of the biometer (Pramer and Bartha, 1965; Pritchard et al., 1992; Mariano et al., 2008). The samples were then incubated in the dark at 30 °C and measured at 1, 2, 4, and 6 days. To measure the CO_2_ produced, the KOH solution was removed from the sidearm of the flask using a 12 mL syringe. The KOH solution was added to 0.2 mL of 1 N barium chloride solution to force any remaining potassium bicarbonate species into potassium carbonate species. The solution was then titrated using 0.05 N hydrochloric acid to a color change, using phenolphthalein as the pH indicator. The sidearm was then refilled with a new KOH solution and placed back in the incubator until the next round of sampling.

(1) $$C_{7}H_{8}+9O_{2}\to 7CO_{2}+4H_{2}O$$

Several experimental controls with un-oxidized soil were run with and without toluene, Haas broth, and microbial inoculums, as shown in Table 1. Biometer tests were also conducted using post oxidation soil and water slurries treated with each oxidant (potassium permanganate, sodium persulfate, sodium percarbonate, and hydrogen peroxide) with and without the addition of toluene. Experiments prepared the slurries and added the toluene as described above. Simple linear regression analysis was performed on CO_2_ production as a function of incubation days to determine the statistical significance of each oxidant treatment.

## 3 Analysis

Gas Chromatography (Wyoming Analytical) measured the toluene concentration. Toluene concentrations were measured using GC-FID (flame ionization detector, Hewlett-Packard 5890 series II) (El-Haj et al., 2000). Eq. (1) above represents the stoichiometric balance for the oxidation of toluene with oxygen to form CO_2_ and water. Eqs. (2) and (3) display the stoichiometric relations for the reaction of CO_2_ with KOH. Finally, Eq. (4) presents the stoichiometry of KOH and HCl's reaction during the titration step. These equations and the required volume/normality of an acid used during titration are employed to calculate the mass of CO_2_ produced. Eq. (5) was used to calculate the volume of the KOH consumed during the reaction.

(2) $$KOH+CO_{2}\to KHCO_{3}$$

(3) $$KOH+KHCO_{3}\to K_{2}CO_{3}+H_{2}O$$

(4) $$KOH+HCl\to H_{2}O+K^{+}+Cl^{-}$$

(5) $$V_{bc}=V_{bi}-\frac{N_{a}*V_{a}}{N_{b}}$$

where, V_bc_ = volume of the KOH consumed (mL), V_bi_ = initial volume of KOH (mL), N_a_ = normality of the titrant (N), V_a_ = volume of titrant (HCL) used to produce a color change (mL), and N_b_ = normality of the KOH solution (N).

## 4 Discussion of results

### 4.1 Biometer control

The biometer control experiments provided the baseline for evaluating the microbial activity change between pre-and post-oxidized soil samples. This data provides the insight to assess changes in microbial activity post-oxidation with each oxidant and statistically assess the significance of CO_2_ produced for each oxidant as a function of incubation times (days) using a 95% confidence interval. The experiments offer a baseline for comparing the post-oxidation effects on microbial activity. The amount of CO_2_ produced by the experiments containing soil, Haas broth, microbes, and toluene and the experiments including soil, Haas broth, and microbes without toluene was the baseline for comparing post-oxidation conditions. Each system shows different levels of CO_2_ production for every experimental state, and as the assumed carbon content for the respective system increases, CO_2_ also increases. Observations could neglect the CO_2_ present in the biometer flask and the CO_2_ produced from the death and utilization of microbial cells.

### 4.2 Effects of permanganate oxidation on microbial activity

Figure 2 shows CO_2_ production as a function of time for each soil samples oxidized with permanganate with/without toluene addition. The figure depicts a direct correlation between the concentration of permanganate and the amount of CO_2_ produced, suggesting that the extent of oxidation increased microbial activity. Table 4 provides the CO_2_ production from pre-to post-oxidation conditions at day six for the cases with and without toluene addition. It also shows the amount of CO_2_ available from the total consumption of toluene by the bacteria. Besides, it shows the actual CO_2_ produced from the addition of toluene for the pre-oxidation control and oxidized soil.

**Figure 2:** Biometer CO_2_ production during post permanganate (KMnO_4_) oxidation (a) without toluene addition and (b) with toluene addition.

**Table 4:** CO_2_ production during pre and post permanganate oxidation.

Sample	CO_2_ production without toluene (μmol)	CO_2_ production with toluene (μmol)	Available CO_2_ from toluene addition (μmol)	Actual CO_2_ production from toluene addition (μmol)
Pre-oxidation control	260.83	303.83	63.00	43.00
KMnO_4_ 0.5 g/L	358.33	453.33	63.00	95.00
KMnO_4_ 1 g/L	475.83	551.67	63.00	75.83
KMnO_4_ 2 g/L	605.00	689.17	63.00	84.17

The samples oxidized with permanganate indicated double the amount of CO_2_ produced than the soil pre-oxidation. In the soils oxidized with permanganate, the microbes made much more CO_2_ than in the pre-oxidation control. Based on the difference between the pre-and post-oxidized soil with toluene, it appears that the microbes were much better able to degrade the toluene in the post-oxidation environment than in the pre-oxidation environment. However, the toluene degradation was not quantitatively measured as a function of time. Experiments adjusted the exact amount of toluene in both instances. The CO_2_ production from the addition of toluene is much higher in the post-oxidation samples than in pre-oxidation controls. The percent increase in CO_2_ output between the pre-and post-oxidized soils was very similar. Nevertheless, the amount of CO_2_ produced from toluene addition is higher than what was added to the system as toluene. The microbes produced as much as twice the amount of CO_2_ from toluene addition in the permanganate oxidized samples than unoxidized soils. Because the addition of toluene is the only difference between the samples with and without toluene for the post-oxidized soils, this indicates that the microbes were better able to utilize toluene as a carbon source following oxidation.

### 4.3 Effects of hydrogen peroxide oxidation on microbial activity

The experimental assessment also evaluated the effects of hydrogen peroxide on enhancing microbial activity in a post-oxidation environment. Figure 3 demonstrates the CO_2_ production of soil samples oxidized with three different hydrogen peroxide concentrations along with the pre-oxidation control. It is interesting to note that the samples oxidized with hydrogen peroxide had a slight increase in microbial activity from the pre-to post-oxidized cases with toluene addition and a slight decrease in microbial activity without toluene addition. Table 5 shows the CO_2_ production from pre-to post-oxidation conditions on day six for the cases with and without toluene addition. It also shows the amount of CO_2_ available from the total consumption of toluene by the bacteria and the actual CO_2_ produced from the addition of toluene for the pre-oxidation control and oxidized soil.

**Figure 3:** Biometer CO_2_ production during post hydrogen peroxide (H_2_O_2_) oxidation (a) without toluene addition and (b) with toluene addition.

**Table 5:** CO_2_ production during pre and post hydrogen peroxide oxidation.

Sample	CO_2_ production without toluene (μmol)	CO_2_ production with toluene (μmol)	Available CO_2_ from toluene addition (μmol)	Actual CO_2_ production from toluene addition (μmol)
Pre-oxidation control	260.83	303.83	63.00	43.00
Hydrogen peroxide 0.46 g/L	193.33	343.33	63.00	150.00
Hydrogen peroxide 0.93 g/L	196.67	350.83	63.00	154.17
Hydrogen peroxide 1.87 g/L	185.00	350.83	63.00	165.83

The concentration of hydrogen peroxide suggested CO_2_ production that was not meaningfully different. Each increase in oxidation had similar CO_2_ output and was consistent both with and without toluene addition. The decrease of the CO_2_ production for the hydrogen-oxidized soil without toluene addition indicates that the oxidation could have a detrimental effect on microbial activity. The difference between the samples with toluene addition and the samples without toluene addition shows more outstanding CO_2_ production from the addition of the toluene post-oxidation. The difference between the samples with and without toluene addition provides that in these oxidized soils, the addition of toluene significantly increased the amount of CO_2_ produced. It indicates that the oxidation with hydrogen peroxide altered the soil to an environment where the microbes, although not as active, were much better able to utilize the toluene. The oxidation of the soil made the conditions less desirable for microbial growth. Yet, with the addition of toluene, the microbes could produce more CO_2_ than can be accounted for from toluene consumption, as shown in Table 5.

### 4.4 Effects of sodium persulfate oxidation on microbial activity

Figure 4 shows the effects of the sodium persulfate treatment. The samples oxidized with toluene show slightly increased CO_2_ production for the post-oxidized soils with toluene addition. Without toluene addition, there is still an increase in CO_2_ output for one oxidant concentration and a slight decrease for the others. The CO_2_ increase rate for the systems without toluene addition post-oxidation is higher than in the pre-oxidation case early in the test. After day one, however, the rate for the oxidized soil plateaus. Table 6 shows the CO_2_ production from pre-to post-oxidation conditions on day six for the cases with and without toluene addition. It also includes the amount of CO_2_ available from the total consumption of toluene by the bacteria and the actual CO_2_ produced from the addition of toluene for the pre-oxidation control and oxidized soil.

**Figure 4:** Biometer CO_2_ production during post sodium persulfate (Na_2_S_2_O_8_) oxidation (a) without toluene addition and (b) with toluene addition.

**Table 6:** CO_2_ production during pre and post sodium persulfate oxidation.

Sample	CO_2_ production without toluene (μmol)	CO_2_ production with toluene (μmol)	Available CO_2_ from toluene addition (μmol)	Actual CO_2_ production from toluene addition (μmol)
Pre-oxidation control	260.83	303.83	63.00	43.00
Sodium persulfate 0.41 g/L	234.17	375.83	63.00	141.67
Sodium persulfate 0.83 g/L	260.83	375.83	63.00	115.00
Sodium persulfate 1.66 g/L	278.33	360.00	63.00	81.67

These samples all revealed significant increases in CO_2_ production with toluene addition in the post-oxidized soils. The gains were all very similar, as oxidation increased CO_2_ production, but the oxidant concentration did not significantly influence the difference. However, the oxidant concentration in the samples without toluene addition exhibited a correlation with the increase or decrease in CO_2_ production from pre-to post-oxidation conditions. The effects of the oxidant concentration on the amount of CO_2_ output are well defined in the case without toluene addition. The difference in CO_2_ production between the samples with/without toluene addition is likely due to the addition of toluene stimulating microbial activity. Thus, the microbes are better at utilizing bioavailable carbon.

The difference in CO_2_ production from toluene supplements was also significant. The post-oxidized soils saw more CO_2_ production increases from the addition of toluene than what experiments observed in the pre-oxidation condition. The CO_2_ production from toluene addition for each system increases as the initial oxidant concentration decreases. The minimal amount of increased CO_2_ production from the addition of toluene is still almost twice as much post-oxidation. The amount of CO_2_ produced from toluene addition is more than can be accounted for from the amount of toluene added. It again indicates that the microbes used carbon provided by toluene to utilize the soil's carbon better.

### 4.5 Effects of sodium percarbonate oxidation on microbial activity

Oxidation with sodium percarbonate resulted in much more CO_2_ production than the other oxidants. However, the CO_2_ production from the microbial activity was not as significant. Figure 5 demonstrates the results. The amount of CO_2_ produced by the systems oxidized with percarbonate with toluene addition was almost three times higher than pre-oxidation. This high increase raised the question of carbonate species being transformed into CO_2_ with the pH buffer's addition. The post-oxidized solution's pH ranged from ∼9.5 to 10.5, and it went ∼7 and 7.5 after pH buffer addition. This decrease in pH was likely responsible for some of the increased CO_2_ production observed. For the soils oxidized with percarbonate, another test was conducted with no microbial addition to the biometer flask to determine the CO_2_ output from only the microbes.

**Figure 5:** Biometer CO_2_ production during post sodium percarbonate (2Na_2_CO_3_.3 H_2_O_2_) oxidation (a) without toluene addition and (b) with toluene addition.

The biometer experiments without microbial addition indicated high amounts of CO_2_ production. This increased production is most likely due to dropping the pH and causing some carbonate species to transform into CO_2_. When CO_2_ produced from the percarbonate oxidized soils without microbial inoculation is ignored, the systems produced far less CO_2_ solely from microbial activity. There is very little difference between the post-oxidized systems without toluene addition both with and without the microbes' addition. Both higher oxidized samples (6.25 g/L and 3.13 g/L) showed the same trend, with the highest initial concentration (6.25 g/L) producing less CO_2_ early. At roughly five days for both conditions, the more oxidized sample begins to make more CO_2_. This trend reinforces just how little of an effect the addition of the microbes had on the production of CO_2_. These percarbonate-oxidized soils altered the soil, thus adversely affecting the microbial activity, showing a high decrease in CO_2_ output from microbial activity. It could be due to the carbon not being transformed into a more bioavailable form.

Table 7 displays the CO_2_ production from pre-to post-oxidation conditions on day six for the cases with and without toluene addition. It also includes the amount of CO_2_ available from the total consumption of toluene by the bacteria and the actual CO_2_ produced from the addition of toluene for the pre-oxidation control and oxidized soil. With toluene addition, there was more CO_2_ production. However, the CO_2_ production in the samples without toluene addition produced minimal CO_2_ from the microbes. This table illustrates just how influenced the CO_2_ production was by merely the percarbonate and buffer reaction. The amount of CO_2_ produced from the microbes in the system was almost non-existent. The sample with toluene addition did show some CO_2_ production generated from the microbial population. When the CO_2_ produced from the system without microbes is removed from the sample, CO_2_ production remaining from the microbes is still far below that of observed pre-oxidation. The carbonate species transforming to CO_2_ controls the CO_2_ production in these samples.

**Table 7:** CO_2_ production during pre and post percarbonate oxidation.

Sample	CO_2_ production without toluene (μmol)	CO_2_ production with toluene (μmol)	Available CO_2_ from toluene addition (μmol)	Actual CO_2_ production from toluene addition (μmol)
Pre-Oxidation Control	260.83	303.83	63.00	43.00
Percarbonate 1.56 g/L	79.17	18.33	63.00	60.83
Percarbonate 3.13 g/L	114.17	35.00	63.00	79.17
Percarbonate 6.25 g/L	104.17	38.33	63.00	65.83

The samples oxidized with percarbonate did not have an overall increase in microbial activity. However, the amount of CO_2_ produced from the addition of toluene was more significant than that found in the pre-oxidized soil samples. As shown in Table 7 above, the CO_2_ increase from the addition of toluene is quite substantial even though the total amount of CO_2_ production is lower than in the pre-oxidation case. Adding toluene to the system resulted in almost twice the amount of CO_2_ output than in the pre-oxidation system from toluene's addition. Again, the amount of CO_2_ produced is higher than what can be accounted for from the addition of toluene.

### 4.6 Comparison of the effects of each oxidant and oxidant concentration

Figure 6 shows the various oxidants plotted together with the pre-oxidation case for each of the three-oxidant equivalents: low, medium, and high. Permanganate oxidation had the greatest effect on microbial activity and the effect increased with concentration. As the concentration of permanganate increased, the difference in CO_2_ production between the pre-and post-oxidized soils also increased, showing a direct correlation. These results suggest that the biodegradability of the natural organic matter in soil increased as the permanganate concentration increased. Each oxidant treatment also showed statistically different levels of CO_2_ production. Hydrogen peroxide and sodium persulfate had very similar impacts on CO_2_ production. These two oxidants showed a slight increase in CO_2_ production over the control samples but the concentration of the oxidant had little impact on CO_2_ production. Sodium percarbonate was the only oxidant to show a deleterious effect. Tables 8 and 9 represent the statistical observation for different oxidant treatments during CO_2_ production with and without toluene.

**Figure 6:** Biometer CO_2_ production for (a) low, (b) medium, and (c) high oxidant concentration with toluene addition.

**Table 8:** Statistical analysis for the CO_2_ production for each oxidant treatment with toluene addition.

Oxidant	Doses	Concentration (g/L)	Toluene condition	Confidence interval	Proportion of variability (R^2^)
Potassium permanganate (KMnO_4_)	High	2.00			0.90
Potassium permanganate (KMnO_4_)	Medium	1.00	Present	95%	0.89
Potassium permanganate (KMnO_4_)	Low	0.50			0.79
Potassium permanganate (KMnO_4_)	Pre-oxidation control	0.00			0.90
Hydrogen peroxide (H_2_O_2_)	High	1.87			0.88
Hydrogen peroxide (H_2_O_2_)	Medium	0.93	Present	95%	0.86
Hydrogen peroxide (H_2_O_2_)	Low	0.46			0.87
Hydrogen peroxide (H_2_O_2_)	Pre-oxidation control	0.00			0.90
Sodium persulfate (Na_2_S_2_O_8_)	High	1.66			0.88
Sodium persulfate (Na_2_S_2_O_8_)	Medium	0.83	Present	95%	0.83
Sodium persulfate (Na_2_S_2_O_8_)	Low	0.41			0.87
Sodium persulfate (Na_2_S_2_O_8_)	Pre-oxidation control	0.00			0.90
Sodium percarbonate (2 Na_2_CO_3_.3 H_2_O_2_)	High	6.25			0.91
Sodium percarbonate (2 Na_2_CO_3_.3 H_2_O_2_)	Medium	3.13	Present	95%	0.90
Sodium percarbonate (2 Na_2_CO_3_.3 H_2_O_2_)	Low	1.56			0.78
Sodium percarbonate (2 Na_2_CO_3_.3 H_2_O_2_)	Pre-oxidation control	0.00			0.90

**Table 9:** Statistical analysis for the CO_2_ production for each oxidant treatment without toluene addition.

Oxidant	Doses	Concentration (g/L)	Toluene condition	Confidence interval	Proportion of variability (R^2^)
Potassium permanganate (KMnO_4_)	High	2.00			0.87
Potassium permanganate (KMnO_4_)	Medium	1.00	Absent	95%	0.81
Potassium permanganate (KMnO_4_)	Low	0.50			0.75
Potassium permanganate (KMnO_4_)	Pre-oxidation control	0.00			0.89
Hydrogen peroxide (H_2_O_2_)	High	1.87			0.61
Hydrogen peroxide (H_2_O_2_)	Medium	0.93	Absent	95%	0.66
Hydrogen peroxide (H_2_O_2_)	Low	0.46			0.87
Hydrogen peroxide (H_2_O_2_)	Pre-oxidation control	0.00			0.89
Sodium persulfate (Na_2_S_2_O_8_)	High	1.66			0.64
Sodium persulfate (Na_2_S_2_O_8_)	Medium	0.83	Absent	95%	0.64
Sodium persulfate (Na_2_S_2_O_8_)	Low	0.41			0.65
Sodium persulfate (Na_2_S_2_O_8_)	Pre-oxidation control	0.00			0.89
Sodium percarbonate (2 Na_2_CO_3_.3 H_2_O_2_)	High	6.25			0.92
Sodium percarbonate (2 Na_2_CO_3_.3 H_2_O_2_)	Medium	3.13	Absent	95%	0.87
Sodium percarbonate (2 Na_2_CO_3_.3 H_2_O_2_)	Low	1.56			0.71
Sodium percarbonate (2 Na_2_CO_3_.3 H_2_O_2_)	Pre-oxidation control	0.00			0.89

The amount of CO_2_ produced from the addition of toluene was frequently higher than the stoichiometric equivalent indicating that the microbes grew better and were more active in the presence of toluene. In each case, the chemical oxidation did not harm the microbe's ability to degrade toluene. In soils oxidized with hydrogen peroxide, the addition of toluene resulted in the most significant increase in CO_2_ production from toluene addition. The amount of CO_2_ produced from toluene was as much as double the amount available from toluene. It suggests that in each post-oxidation case, the microbes also better utilized the toluene than in the pre-oxidation control. The oxidation of NOM likely forced the microbes to use toluene as some of the available carbon was not bioavailable. It also may indicate that a contaminant would be better-degraded post-oxidation even if the overall microbial activity decreased. A comparison of the CO_2_ produced from the toluene added is shown as the amount higher and lower than 63 μmol of CO_2_, which is the amount of CO_2_ available from toluene's addition.

## 5 Conclusions

Oxidation with permanganate revealed the highest increase in microbial activity post oxidation based on CO_2_ production, both with and without the toluene's addition. The permanganate oxidized soils also indicated the strongest direct correlation between increasing oxidant concentration and increased CO_2_ production. Permanganate had the most significant effect on reducing NOD and exhibited the greatest increase in CO_2_ production. It is likely that the soil oxidized by permanganate was more suitable for overall microbial activity as a result of previously unavailable organic carbon being oxidized into more biodegradable forms. Unlike permanganate, oxidation with hydrogen peroxide did not show a strong direct correlation between increasing oxidant concentration and increased CO_2_ production. Although hydrogen peroxide oxidation did show an increase in microbial activity following toluene addition it decreased without toluene from the pre-oxidation control. The addition of toluene likely stimulated increased microbial growth and the microbes utilized the carbon in the soil at a faster rate.

Sodium persulfate oxidation showed increased microbial activity post oxidation after toluene's addition and decreased without toluene. There was no correlation between initial oxidant concentration and CO_2_ production increase. The addition of toluene stimulated CO_2_ production and showed more CO_2_ than what is available from toluene. The post-oxidized system using persulfate was more suitable for microbial activity with toluene and less convenient without toluene. The post-oxidation environment was better for natural attenuation. The oxidant sodium percarbonate showed the only adverse effects post-oxidation. The addition of toluene stimulated microbial growth in the system, allowing microbes to utilize the bioavailable carbon in the soil more quickly. It likely increased CO_2_ production from toluene compared to the available CO_2_ from the toluene addition. The system, however, was overall less suited for microbial activity.

The oxidation with potassium permanganate, hydrogen peroxide, and sodium persulfate resulted in an increased or statistically unchanged microbial activity. The oxidation with sodium percarbonate showed the only harmful effects on microbial activity. Regardless of the oxidant, oxidation resulted in more CO_2_ production from the bacteria *Pseudomonas putida F1* than can be accounted for by the addition of toluene alone. It also indicates that microbes more completely degraded the toluene during post-oxidation. The microbes used toluene and bioavailable CO_2_ more quickly during post oxidation. It suggests that soil's carbon was more bioavailable in the post-oxidized soil. It indicates that the microbes used the toluene and efficiently consumed the bioavailable carbon in the oxidized system. Although there was a direct correlation between oxidant concentration and PCOD removal in soil, permanganate was the only oxidant that showed a correlation between PCOD removal and microbial activity. It would appear that permanganate oxidation of the natural organic matter in soil may actually result in greater bioavailability thus stimulating microbial growth.

## Declarations

### Author contribution statement

Mohan B. Dangi & Michael A. Urynowicz: Conceived and designed the experiments; Analyzed and interpreted the data; Contributed reagents, materials, analysis tools or data; Wrote the paper.

Christopher L. Schultz: Conceived and designed the experiments; Performed the experiments; Analyzed and interpreted the data; Contributed reagents, materials, analysis tools or data.

Samir Budhathoki: Analyzed and interpreted the data; Contributed reagents, materials, analysis tools or data; Wrote the paper.

Sadikshya R. Dangi: Analyzed and interpreted the data; Wrote the paper.

### Funding statement

This research did not receive any specific grant from funding agencies in the public, commercial, or not-for-profit sectors.

### Data availability statement

Data will be made available on request.

### Declaration of interests statement

The authors declare no conflict of interest.

### Additional information

No additional information is available for this paper.

## References

[bib1] Abuhamed T., Bayraktar E., Mehmetoǧlu T., Mehmetoǧlu Ü. (2004). Kinetics model for growth of Pseudomonas putida F1 during benzene, toluene and phenol biodegradation. Process Biochem..

[bib2] Apul O.G., Dahlen P., Delgado A.G., Sharif F., Westerhoff P. (2016). Treatment of heavy, long-chain petroleum-hydrocarbon impacted soils using chemical oxidation. J. Environ. Eng..

[bib3] Atalay S., Ersöz G. (2016).

[bib5] Bolade O.P., Adeniyi K.O., Williams A.B., Benson N.U. (2021). Remediation and optimization of petroleum hydrocarbons degradation in contaminated water using alkaline activated persulphate. J. Environ. Chem. Eng..

[bib6] Bordel S., Muñoz R., Díaz L.F., Villaverde S. (2007). New insights on toluene biodegradation by Pseudomonas putida F1: influence of pollutant concentration and excreted metabolites. Appl. Microbiol. Biotechnol..

[bib7] Buthiyappan A., Abdul Aziz A.R., Wan Daud W.M.A. (2016). Recent advances and prospects of catalytic advanced oxidation process in treating textile effluents. Rev. Chem. Eng..

[bib8] Cuerda-Correa E.M., Alexandre-Franco M.F., Fernández-González C. (2020). Advanced oxidation processes for the removal of antibiotics from water. An overview. Water (Switzerland).

[bib9] Cajal-Mariñosa P., De La Calle R.G., Rivas F.J., Tuhkanen T. (2012). Impacts of changing operational parameters of in situ chemical oxidation (ISCO) on removal of aged PAHs from soil. J. Adv. Oxid. Technol..

[bib10] Chicca I., Becarelli S., Dartiahl C., La China S., De Kievit T., Petroni G., Di Gregorio S., Levin D.B. (2020). Degradation of BTEX mixture by a new Pseudomonas putida strain: role of the quorum sensing in the modulation of the upper BTEX oxidative pathway. Environ. Sci. Pollut. Control Ser..

[bib11] Cui H., Gu X., Lu S., Fu X., Zhang X., Fu G.Y., Qiu Z., Sui Q. (2017). Degradation of ethylbenzene in aqueous solution by sodium percarbonate activated with EDDS–Fe(III) complex. Chem. Eng. J..

[bib12] Danish M., Gu X., Lu S., Ahmad A., Naqvi M., Farooq U., Zhang X., Fu X., Miao Z., Xue Y. (2017). Efficient transformation of trichloroethylene activated through sodium percarbonate using heterogeneous zeolite supported nano zero valent iron-copper bimetallic composite. Chem. Eng. J..

[bib13] Devi P., Das U., Dalai A.K. (2016). In-situ chemical oxidation: principle and applications of peroxide and persulfate treatments in wastewater systems. Sci. Total Environ..

[bib14] Díaz L.F., Muñoz R., Bordel S., Villaverde S. (2008). Toluene biodegradation by Pseudomonas putida F1: targeting culture stability in long-term operation. Biodegradation.

[bib15] El-Haj B.M., Al-Amri A.M., Hassan M.H., Bin-Khadem R.K., Al-Hadi A.A. (2000). A GC-MS method for the detection of toluene and ethylbenzene in volatile substance abuse. J. Anal. Toxicol..

[bib16] Fu X., Gu X., Lu S., Miao Z., Xu M., Zhang X., Qiu Z., Sui Q. (2015). Benzene depletion by Fe2+-catalyzed sodium percarbonate in aqueous solution. Chem. Eng. J..

[bib17] Hamidi A.A., Salem S.A. (2015). Performance of combined ozone and Fenton process in treating different leachate concentrations. Sustain. Energy Environ..

[bib18] Huang Z., Liu F., Urynowicz M.A., Basile F., Guo H., Chen L., Fallgren P.H., Jin S. (2018). Coal-derived compounds and their potential impact on groundwater quality during coalbed methane production. Environ. Geochem. Health.

[bib19] Huang Z., Urynowicz M.A., Colberg P.J.S. (2013). Bioassay of chemically treated subbituminous coal derivatives using Pseudomonas putida F1. Int. J. Coal Geol..

[bib20] Huang Z., Urynowicz M.A., Colberg P.J.S. (2013). Stimulation of biogenic methane generation in coal samples following chemical treatment with potassium permanganate. Fuel.

[bib21] Huling S.G., Pivetz B.E. (2002). Engineering issues. Fire Int..

[bib22] Hyat M.A. (1989).

[bib23] Interscience L.M. (1910). Books received. J. Soc. Chem. Indust..

[bib24] Khodaveisi J., Banejad H., Afkhami A., Olyaie E., Lashgari S., Dashti R. (2011). Synthesis of calcium peroxide nanoparticles as an innovative reagent for in situ chemical oxidation. J. Hazard Mater..

[bib25] King N.S., Luster-Teasley S., Clark C.J. (2021). Preliminary analyses of controlled release of potassium permanganate encapsulated in polycaprolactone. J. Water Resour. Protect..

[bib26] Li X.D., Schwartz F.W. (2004). DNAPL remediation with in situ chemical oxidation using potassium permanganatey. Part I. Mineralogy of Mn oxide and its dissolution in organic acids. J. Contam. Hydrol..

[bib27] Liang C., Su H.W. (2009). Identification of sulfate and hydroxyl radicals in thermally activated persulfate. Ind. Eng. Chem. Res..

[bib28] Liu H., Bruton T.A., Doyle F.M., Sedlak D.L. (2014). In situ chemical oxidation of contaminated groundwater by persulfate: decomposition by Fe(III)- and Mn(IV)-containing oxides and aquifer materials. Environ. Sci. Technol..

[bib29] Ma J., Xia X., Ma Y., Luo Y., Zhong Y. (2018). Stability of dissolved percarbonate and its implications for groundwater remediation. Chemosphere.

[bib30] Mariano A.P., Tomasella R.C., De Oliveira L.M., Contiero J., De Angelis D.D.F. (2008). Biodegradability of diesel and biodiesel blends. Afr. J. Biotechnol..

[bib31] Miao Z., Gu X., Lu S., Brusseau M.L., Zhang X., Fu X., Danish M., Qiu Z., Sui Q. (2015). Enhancement effects of chelating agents on the degradation of tetrachloroethene in Fe(III) catalyzed percarbonate system. Chem. Eng. J..

[bib32] Miao Z., Gu X., Lu S., Dionysiou D.D., Al-Abed S.R., Zang X., Wu X., Qiu Z., Sui Q., Danish M. (2015). Mechanism of PCE oxidation by percarbonate in a chelated Fe(II)-based catalyzed system. Chem. Eng. J..

[bib33] Miao Z., Gu X., Lu S., Zang X., Wu X., Xu M., Ndong L.B.B., Qiu Z., Sui Q., Fu G.Y. (2015). Perchloroethylene (PCE) oxidation by percarbonate in Fe2+-catalyzed aqueous solution: PCE performance and its removal mechanism. Chemosphere.

[bib34] Pal D.B., Giri D.D. (2021). Sustainable Environmental Clean-Up.

[bib35] Pardieck D.L., Bouwer E.J., Stone A.T. (1992). Hydrogen peroxide use to increase oxidant capacity for in situ bioremediation of contaminated soils and aquifers: a review. J. Contam. Hydrol..

[bib36] Pramer D., Bartha R. (1965). Features of flask and method for measurement of the persistence and biological effects of pesticides in soil. Soil Sci..

[bib37] Pritchard P.H., Mueller J.G., Rogers J.C., Kremer F.V., Glaser J.A. (1992). Oil spill bioremediation: experiences, lessons and results from the Exxon Valdez oil spill in Alaska. Biodegradation.

[bib38] Reardon K.F., Mosteller D.C., Bull Rogers J.D. (2000). Biodegradation kinetics of benzene, toluene, and phenol as single and mixed substrates for Pseudomonas putida F1. Biotechnol. Bioeng..

[bib39] Robledo-Ortíz J.R., Ramírez-Arreola D.E., Pérez-Fonseca A.A., Gómez C., González-Reynoso O., Ramos-Quirarte J., González-Núñez R. (2011). Benzene, toluene, and o-xylene degradation by free and immobilized P. putida F1 of postconsumer agave-fiber/polymer foamed composites. Int. Biodeterior. Biodegrad..

[bib40] Romero A., Santos A., Vicente F., Rodriguez S., Lafuente A.L. (2009). In situ oxidation remediation technologies: kinetic of hydrogen peroxide decomposition on soil organic matter. J. Hazard Mater..

[bib41] Sutton N.B., Grotenhuis J.T.C., Langenhoff A.A.M., Rijnaarts H.H.M. (2011). Efforts to improve coupled in situ chemical oxidation with bioremediation: a review of optimization strategies. J. Soils Sediments.

[bib42] Timmis K.N. (2002). Pseudomonas putida : a cosmopolitan. Environ. Microbiol..

[bib43] Tsitonaki A., Petri B., Crimi M., Mosbk H., Siegrist R.L., Bjerg P.L. (2010). In situ chemical oxidation of contaminated soil and groundwater using persulfate: a review. Crit. Rev. Environ. Sci. Technol..

[bib44] Urynowicz M.A. (2007). In situ chemical oxidation with permanganate: assessing the competitive interactions between target and nontarget compounds. Soil Sediment Contam..

[bib45] Urynowicz M.A., Balu B., Udayasankar U. (2008). Kinetics of natural oxidant demand by permanganate in aquifer solids. J. Contam. Hydrol..

[bib46] Viisimaa M., Goi A. (2014). Use of hydrogen peroxide and percarbonate to treat chlorinated aromatic hydrocarbon-contaminated soil. J. Environ. Eng. Landsc. Manag..

[bib47] Waldemer R.H., Tratnyek P.G. (2006). Kinetics of contaminant degradation by permanganate. Environ. Sci. Technol..

[bib48] Xu X.R., Li X.Z. (2010). Degradation of azo dye Orange G in aqueous solutions by persulfate with ferrous ion. Separ. Purif. Technol..

[bib49] Xu X., Thomson N.R. (2008). Estimation of the maximum consumption of permanganate by aquifer solids using a modified chemical oxygen demand test. J. Environ. Eng..

